The article "Building a richer understanding of diversity through causally consistent evenness measures" was retracted in 2020. Reasons: concerns about the data; concerns about the results or conclusions.

# Building a richer understanding of diversity through causally consistent evenness measures

**DOI:** 10.1002/ece3.6353

**Published:** 2020-05-26

**Authors:** Kawika Pierson

**Affiliations:** ^1^ Atkinson Graduate School of Management Willamette University Salem OR USA

**Keywords:** causal consistency, diversity, evenness, evenness–unevenness index, percent richness

## Abstract

Causally consistent evenness measures can only be changed when the populations they refer to change. This novel property is deeply important for making causal inferences, and yet every prominent evenness measure is not causally consistent. This paper proposes a family of causally consistent evenness measures, and while any evenness measure can be made to be causally consistent, the family I introduce has the added benefit of a straightforward interpretation as a percentage evenness. I go on to illustrate the performance of these measures, and demonstrate the importance of causal consistency not only for causal inference but also for correctly reflecting the evenness of ecological communities. I also present several alternative transformations of my preferred measures, which work to address potential critiques in advance, communicate evenness to nontechnical audiences, and connect my work to more familiar ecological indicators.

## Graphical abstract

Causal consistency is a novel and important requirement for an evenness measure because it ensures that the only way for evenness to change is through changes to species abundances. We discuss the importance of causal consistency and provide several causally consistent evenness measures that are also easy to interpret as percentages.

## 1 INTRODUCTION

It is well accepted that diversity is a concept composed of two related facets: richness, which reflects the effective number of species present in a community, and evenness, which is about how uniformly that community is divided (Hill, 1973). While ecologists have reached a consensus around the use of the Hill numbers, also known as diversities of order q, to measure richness (Jost, 2006), the available evenness measures have proven consistently less appealing (Kvålseth, 2015; Smith & Wilson, 1996; Tuomisto, 2012).

Even after decades of work on the measurement of diversity, ecologists and biologists still regularly make difficult trade‐offs whenever they reach for a measure of evenness, since common choices such as the Gini index (Gini 1912; Stensrud & Valberg, 2017; Wittebolle et al., 2009), Hill evenness (Tuomisto, 2012), or Pielou's J (Ehsani et al., 2018; Rohr et al., 2016) are not entirely convincing. These challenges around measuring the concept have not stopped researchers from recognizing the importance of evenness for regulating and impacting many different ecological processes, however. Whether for its role in extinctions (Rohr et al., 2016), the ability of a community to resist environmental stress (Wittebolle et al., 2009), or the carbon absorption capacity of a forest (Shirima, Totland, Munishi, & Moe, 2015), the role of evenness in understanding ecological dynamics, and thus the need for an easy to understand measure of evenness, has never been so clear.

This paper presents a new family of easily interpretable measures of evenness, which I call ^q^D_E_ or q‐order percentage evenness measures. This family performs well as a measure of evenness, since it is quite similar in structure to a family of measures discussed in Chao and Ricotta (2019). Where ^q^D_E_ clearly outperforms existing measures however is in the fact that ^q^D_E_ is causally consistent.

I define causal consistency to mean that the only way to change the value that a measure calculates for a given community is to change the abundances of the individuals in that community. All existing evenness measures fail this test for a narrow, but scientifically important, fact pattern: changes in the number of species considered by the study. The ecological dynamics of an isolated community should never depend on whether a different community includes a rare species, or worse, whether investigators decide to include some set of species in their research design.

The fact that my evenness measures are the first causally consistent measures reported is not a result of some clever mathematical trick. Instead, their causal consistency comes from a conceptual shift in how species richness is used in their calculation. By focusing only on the abundances of species that actually exist in a given population, the family of evenness measures ^q^D_E_ is able to better accentuate the impact of rare species on evenness, better reflect the actual evenness of the species which are present, and better support causal inference by establishing itself as causally consistent.

I go on to describe two additional families of measures that can provide other perspectives on a community's evenness. The evenness–unevenness index, ^q^EU, stretches ^q^D_E_ to extend the measure's range from −1 to 1, so that the midpoint of ^q^D_E_ corresponds to a conceptual break between relatively even communities and relatively uneven ones. Another family of measures ^q^P_E_ overemphasizes the importance of rare species for the calculation of evenness, and are also replication‐invariant, a controversial property of evenness measures that some scholars desire.

Together these simple, but novel, measures of evenness have the potential to immediately enhance our understanding of a vast body of work in ecology and the biological sciences, and will give future researchers a roadmap for deploying measures of evenness alongside measures of richness so that we can bring a truly binocular perspective to this two‐dimensional topic.

## 2 EXISTING EVENNESS MEASURES

All measures of diversity and evenness take as their input a list of species proportions p_s_. To construct these proportions, first list the S species that have been identified across all of the plots being studied. Next, count the abundance of each species at each plot. Last, use these abundances to calculate the S proportions p_s_ as the fraction of the community belonging to each species at each plot. In addition, define K for a plot to be the number of species from the list S that have nonzero abundances at that plot.

The two most popular measures of evenness share common roots in the seminal work of Shannon (1948) and Simpson (1949) on entropy and diversity. These foundational ideas were directly applied to the study of evenness by Pielou who developed a measure J (Heip, 1974; Pielou, 1975) that is a simple transformation of Shannon entropy and is calculated as:

$$J=\frac{-\sum_{s=1}^{S}p_{s}\cdot \ln\left(p_{s}\right)}{\ln\left(S\right)}$$

At the same time, Hill (1973) was developing an approach to evenness that was derived from his measures of species richness. This family of richness measures, commonly called the Hill numbers (Chao et al., 2014; Hill, 1973), but which I label ^q^D_R_ in order to emphasize that they are richness‐focused diversity measures, is calculated from the list of proportions p_s_ as:

$${\;}^{q}D_{R}\equiv \left\{\begin{array}{ccc} \frac{1}{{\left(\sum_{s=1}^{S}p_{s}^{q}\right)}^{1/\left(q-1\right)}} & , & \;q\neq 1\\ \exp\left[-\sum_{s=1}^{S}p_{s}\cdot \ln\left(p_{s}\right)\right] & , & \;q=1\\ \frac{1}{\mathrm{Max}(p_{s})} & , & \;q=\infty \\ K & , & \;q=0 \end{array}\right.$$

The construction of this measure as a “family” gives the user the option to choose an order *q* from the positive integers. Each *q* is a different Hill number, but they all measure the richness of ecological communities since they can all be interpreted as measures of the effective number of species present in a community. For example, if you apply any ^q^D_R_ to a community with *N* evenly distributed species the answer will always equal *N*, and doubling the number of species for an arbitrary community by dividing every species exactly in half will always precisely double ^q^D_R_ (Jost, 2006).

While some use the term richness strictly to mean the count of the number of species present (K or ^0^D_R_), all ^q^D_R_ are richness‐focused measures, even if they are not pure richness. The order *q* modulates the importance of evenness in determining the effective number of species reported by ^q^D_R_. For *q* = 0, no evenness information is considered, and as *q* gets larger, so does the importance of evenness in determining the value of ^q^D_R_. Because of this property, Hill (1973) proposed scaling two members of ^q^D_R_ as a way of expressing evenness. Specifically, he suggested:

$$E_{2,1}={\;}^{2}D_{R}/{\;}^{1}D_{R}$$

or

$$E_{q,S}={\;}^{q}D_{R}/S$$

This approach, sometimes called Hill evenness, and Pielou's J are the two most influential evenness measures, and both are widely employed in practice (Morris et al., 2014; Ricotta, 2017). There are many other measures that have been suggested however, so many in fact that a complete exposition of them here is impractical. Broadly though, they take one of two approaches to improving on Pielou's J and Hill evenness: either employing considerably more complicated mathematical functions (Camargo, 2008; Nijssen, Rousseau, & Van Hecke, 1998; Smith & Wilson, 1996) or cleverly transforming other diversity measures (Chao & Ricotta, 2019; Kvålseth, 2015).

Since complicated mathematical expressions run counter to my stated goal of delivering a simple to interpret measure, I will not discuss that group further. Instead, I will turn my attention to the second approach. Specifically, notice how the Hill numbers ^q^D_R_ can be reciprocated in order to calculate a family of concentration measures which I call ^q^C:

$${\;}^{q}C\equiv \left\{\begin{array}{ccc} {\left(\sum_{s=1}^{S}p_{s}^{q}\right)}^{1/\left(q-1\right)} & , & \;q\neq 1\\ \exp\left[\sum_{s=1}^{S}p_{s}\cdot \ln\left(p_{s}\right)\right] & , & \;q=1\\ \mathrm{Max}(p_{s}) & , & \;q=\infty \\ \frac{1}{K} & , & \;q=0 \end{array}\right.$$

A clever transformation of ^q^C is one of the families of evenness measures discussed by Chao and Ricotta (2019). This “anti‐concentration”‐based evenness measure ^q^C_E_ first takes the additive inverse of concentration and then scales the result by its maximum value, which depends on the number of species S present in the study:

$${\;}^{q}C_{E}\equiv \frac{1-{\;}^{q}C}{1-\left(1/S\right)}=\left\{\begin{array}{ccc} \frac{1-{\left(\sum_{s=1}^{S}p_{s}^{q}\right)}^{1/\left(q-1\right)}}{1-\left(1/S\right)} & , & \;q\neq 1\\ \frac{1-\exp\left[\sum_{s=1}^{S}p_{s}\cdot \ln\left(p_{s}\right)\right]}{1-\left(1/S\right)} & , & \;q=1\\ \frac{1-\mathrm{Max}(p_{s})}{1-\left(1/S\right)} & , & \;q=\infty \\ \frac{1-\left(1/K\right)}{1-\left(1/S\right)} & , & \;q=0 \end{array}\right.$$

If you choose q equal to 2, then ^2^C_E_ is equivalent to the transformation of Simpson dominance (Simpson, 1949) noted by Pielou (and Smith & Wilson, 1996), but otherwise, this approach to measuring evenness was first proposed by Chao and Ricotta (2019). While this is only one of a number of measures that they discuss, I believe that this measure has a simple, persuasive interpretation which I will discuss later, and so I feel it is important to highlight here.

## 3 DEBATED REQUIREMENTS OF AN EVENNESS MEASURE

As the number of papers discussing evenness grew, so did the number of proposed measures. In response to this proliferation, an effort began to lay out a set of requirements that a good measure of evenness should satisfy. An early, influential example is Smith and Wilson’s (1996) “Consumer's Guide to Evenness,” which gives a number of requirements. They argue that an evenness measure should be independent of species richness, decrease from marginally reducing the least abundant species, decrease from the addition of a rare species, and reach a maximum value of 1 for perfectly even abundances, along with a number of other suggestions. While no evenness measure satisfies all of their requirements, their requirement that a measure of evenness should be independent of species richness has been the most hotly debated.

One reason for this tension is that, as Jost (2010) persuasively argues, it is mathematically impossible to decompose diversity into independent evenness and richness components. So, rather than achieving true independence it has become common to adopt a term like “unrelatedness” as the goal (Chao, Chiu, & Hsieh, 2012). This call for an evenness measure to be unrelated to species richness is one of the core arguments against using Hill evenness. A measure that is the ratio of two richness measures seems unconvincing as a measure of evenness because it depends too much on the richness of the community.

In contrast, Tuomisto (2012) is a strong proponent of using a version of Hill evenness, because they argue that an evenness measure should have a property called “replication invariance.” This property says that doubling the size of a population by replicating its individuals and then counting those additions as members of new species should leave a measure of evenness unchanged. This suggestion has not been well received, however. Many scholars of evenness (Chao & Ricotta, 2019; Kvålseth, 2015) dismiss the call for replication invariance because replication introduces new species with equal populations to all of the existing species, and so it intuitively should increase evenness, not keep evenness constant. They view the desire for replication invariance as the result of overapplying a richness‐based view to the measurement of evenness.

Kvålseth (2015) suggests that an evenness measure should exhibit a property called Schur‐concavity. This property emerges from an attempt to formally define our expectations for the relative evenness of two lists of proportions. Consider two lists of proportions p_s_1 and p_s_2, each arranged in decreasing order. If the sum of the N largest proportions in p_s_1 is larger than the sum of the *N* largest proportions in p_s_2 for all *N* < S, then p_s_1 is said to majorize p_s_2. Kvålseth (2015) argues that any list that majorizes another must be less even, and so a valid evenness measure will calculate that the evenness of p_s_1 is less than the evenness of p_s_2. This property is called Schur‐concavity.

A weakness in this approach is that the Kvålseth (2015) definition of Schur‐concavity allows some proportions in the vectors to take a value of zero. More recent work by Chao and Ricotta (2019) correctly remarks that “strict” Schur‐concavity should only apply when the actual number of species in each list, *K*, is equal. To understand why, note, as they do, that a community with two species perfectly dividing its population would have proportions p_s_1 = (0.5, 0.5) and would be maximally even. Yet if there were any plot with more than two species, its proportions would often be majorized by p_s_1, since the sum of the two largest elements of p_s_1 would equal 1. That second plot would be less than maximally even in almost all cases however, leading to a contradiction. Thus, Schur‐concavity should only be required when the number of species in each plot, K, is equal, since our intuition about evenness runs counter to this example.

Most recently, Chao and Ricotta (2019) propose the following list of requirements for an evenness measure: Transfers of individuals from more abundant species to less abundant species should increase evenness (the principle of transfer), the measure should be continuous and invariant under changes in the ordering of proportions, the introduction of a rare species should not cause the calculated evenness to increase, the measure should take a fixed range regardless of the values taken by richness‐focused diversity measures ^q^D_R_, evenness should not be impacted by the units used, Schur‐concavity should hold when K is fixed, and evenness should increase under a replication of species. All of the measures they discuss, including the one I call ^q^C_E_, adhere to these requirements.

## 4 CAUSAL CONSISTENCY

The main contribution of this paper is to propose a new property called causal consistency that any evenness measure, or indeed any measure of diversity, should have. A diversity measure can be said to be causally consistent if the only way to change the value calculated by the measure for a given plot is by changing the species abundances at that plot. Logically, if we wish to build causal inferences around the role of evenness in ecological communities, then evenness should only change when abundances change. If the value of a measure of evenness is impacted by changes to research designs or the abundances of causally isolated communities, then that measure of evenness is not capturing something intrinsic to the community being measured.

In order to understand why this is important, consider a simple example. Imagine two plots, 1 and 2, which are remote from each other. Say that you begin with two possible species, and that your communities at 1 and 2 each have 50% of their individuals coming from each species, such that p_s_1 = p_s_2 = (0.5, 0.5). Both plots are perfectly even in this case, and most evenness metrics will return a value of 100% for both p_s_1 and p_s_2.

Now imagine that you wanted to test a hypothesis about the impact that a third, perhaps invasive species, has on some important ecological outcome. One potential approach might be to experimentally introduce a few individuals of that species into one of the plots, say plot 1, and to treat the other community as a control. This action directly manipulates the evenness of community 1, and so you would expect measures of evenness to decrease for that community. Most existing measures perform well here since p_s_1 has become considerably less even, perhaps now equaling (0.49, 0.49, 0.02).

Causal consistency is about recognizing that nothing has changed for community 2, and so its measure of evenness should remain 100% even though its list of proportions has changed to (0.5, 0.5, 0). Because the experimental setup is predicated on the idea that there is no plausible causal pathway for the rare species at plot 1 to impact the ecology of plot 2, your measure of evenness must also be consistent with that understanding. Unfortunately, existing measures of evenness would universally rank (0.5, 0.5, 0) as *less* even than (0.49, 0.49, 0.02), because the former has no individuals of the third species.

The central reason that all existing *evenness* measures fail this test is because they do not properly distinguish between the number of possible species considered by the study, S, and the specific number of species present in a particular location, K. The richness‐focused Hill numbers ^q^D_R_ are all causally consistent, since they mechanically ignore any species abundance counts of zero. Perhaps because causal consistency was never an issue in the study of richness, or perhaps because of the subtlety of this concept, this paper is the first to recognize that evenness measures must also exhibit causal consistency.

## 5 A CAUSALLY CONSISTENT EVENNESS MEASURE

Any evenness measure can be adjusted to become causally consistent if it correctly distinguishes between K and S. In order to illustrate how this can be achieved, I create a causally consistent version of ^q^C_E_ from Chao and Ricotta (2019). I choose this measure because, with a slight change to the way it is presented, it is easy to view ^q^C_E_ as a percentage evenness. This is important to emphasize in order to give my measure of evenness a high level of interpretive clarity.

My measure, which I call ^q^D_E_, is, like ^q^C_E_, a fraction. The numerator is the additive inverse of the concentration measure ^q^C, and the denominator scales 1−^q^C by the value we would expect 1‐^q^C to take in a perfectly equal community with K species. This measure is causally consistent because I scale its value using the actual number of species at each plot, K, rather than the total number of species between all plots, S. Specifically, ^q^D_E_ is calculated as:

$$\begin{array}{c} {\;}^{q}D_{E}\equiv \frac{1-{\;}^{q}C}{\left(K-1\right)/K}\\ =\left\{\begin{array}{ccc} \frac{K}{\left(K-1\right)}\cdot \left[1-{\left(\sum_{s=1}^{S}p_{s}^{q}\right)}^{\frac{1}{q-1}}\right] & , & \;q\neq 1\;\;\mathrm{and}\;\;K\neq 1\\ \frac{K}{\left(K-1\right)}\cdot \left\{1-\exp\left[\sum_{s=1}^{S}p_{s}\cdot \ln\left(p_{s}\right)\right]\right\} & , & \;q=1\;\;\mathrm{and}\;\;K\neq 1\\ \frac{K}{\left(K-1\right)}\cdot \left[1-\mathrm{Max}(p_{s})\right] & , & \;q=\infty \\ 1 & , & \;q=0\;\mathrm{or}\;K=1 \end{array}\right. \end{array}$$

This conceptualization of ^q^D_E_ owes a great debt to Hurlburt's probability of interspecific encounter (Hurlbert, 1971), which is sometimes mentioned in discussions of evenness because of its interpretation as a probability (Olszewski, 2004). The probability of interspecific encounter's probabilistic interpretation is that it is the chance that any two random draws from the population will produce two individuals of different species. Rather than settle for an evenness measure that is most easily described as the sum of multiple simultaneous conditional probabilities however, ^q^D_E_ acknowledges the central role that the actual number of species present in a specific community plays in the way we should think about the evenness of those K species.

Mathematically, consider the case where *q* equals 2 and ^2^D_E_ is a scaled version of the probability of interspecific encounter. Any perfectly even community will always produce a probability of interspecific encounter equal to (K−1)/K because no matter what the first draw produces the second draw will always have K−1 equally sized species that are different from the first. Dividing the probability of interspecific encounter by (K−1)/K then will rescale the measure so that it is expressed as a percentage of its maximum value. This scaling gives the index a value of 1 for any perfectly even community and a value arbitrarily close to 0 for any highly uneven one, suggesting that we can interpret it as percentage evenness or, more operationally, as a percentage of the maximum probability of interspecific encounter possible given the value of K observed.

Using the plot‐specific value K, rather than the absolute standard S, allows us to compare evenness consistently across communities when the value of K changes. The absolute standard used in ^q^C_E_ assumes that every species must exist in every plot for that plot to be truly even. When Chao and Ricotta (2019) discuss how Schur‐concavity is only valid for cases where the number of species is equal, they come very close to seeing this insight, yet all of the measures they propose, including ^q^C_E_, are causally inconsistent because they all punish potentially even communities for not having members of every species present across all plots.

This distinction is not just about causal inference, it matters for measuring evenness as well. The values calculated by ^q^D_E_ demonstrate how the introduction of a rare species decreases evenness more for a low‐richness community than it does for a high‐richness community. Consider a simple case of two perfectly even communities. Starting with two species of 500 individuals each and adding a single individual of a third species will drastically reduce the evenness of that community, because adding this species increases the maximum possible probability of interspecific encounter from 1/2 to 2/3. On the other hand, starting with eight species of 125 individuals each and adding a single individual of a ninth species only moves the maximum probability of interspecific encounter from 7/8 to 8/9, and so the *percentage* evenness of the high‐richness community has been reduced by considerably less than the percentage evenness of the low‐richness community from the addition of one species (Heip, Herman, & Soetaert, 1998).

Because this family of measures is constructed using ^q^C, the order *q* controls the importance of richness in determining the evenness calculated, mirroring the way that this same term controls the importance of evenness in determining the richness calculated by the Hill numbers. A larger value of q makes richness more influential in the measured value of ^q^D_E_.

Because the family ^q^D_E_ is very similar to the family ^q^C_E_ discussed in Chao and Ricotta (2019), it performs very well along all of the dimensions typically used to evaluate evenness measures (Chao & Ricotta, 2019; Kvålseth, 2015; Smith & Wilson, 1996). In my opinion though, the ease of interpreting ^q^D_E_ as a percentage evenness recommends it over the many alternative measures. I will illustrate ^q^D_E_’s performance and simple interpretation after I introduce two additional measures that may be of interest.

## 6 ADDITIONAL EVENNESS MEASURES

If we are willing to relax the assumption that an evenness measure must be bounded between zero and one, then a linear transformation of ^q^D_E_ that I call the evenness–unevenness index, or ^q^EU, may be an interesting alternative:

$$\begin{array}{c} {\;}^{q}EU\equiv \left(2\cdot^{q}D_{E}\right)-1\\ =\left\{\begin{array}{ccc} \;2\cdot \left\{\frac{K}{\left(K-1\right)}\cdot \left[1-{\left(\sum_{s=1}^{S}p_{s}^{q}\right)}^{\frac{1}{q-1}}\right]\right\}-1 & , & \;q\neq 1\;\;\mathrm{and}\;\;K\neq 1\\ 2\cdot \left(\frac{K}{\left(K-1\right)}\cdot \left\{1-\exp\left[\sum_{s=1}^{S}p_{s}\cdot \ln\left(p_{s}\right)\right]\right\}\right)-1 & , & \;q=1\;\;\mathrm{and}\;\;K\neq 1\\ 1 & , & \;K=1\\ 2\cdot \left[\frac{K}{\left(K-1\right)}\cdot \left[1-\mathrm{Max}(p_{s})\right]\right]-1 & , & \;q=0 \end{array}\right. \end{array}$$

^q^EU contains the same information as ^q^D_E_, but because it ranges from −1 to 1, its values communicate either percentage evenness or percentage unevenness. This behavior can improve the correspondence between evenness measures and a nontechnical understanding of the concept. By assigning any community with a ^q^D_E_ of 50% to a ^q^EU of 0%, it lessens the natural tendency to look at a “40% even” community and remark that it does not look particularly even. ^q^EU communicates the fact that a community with a ^q^D_E_ of 40% really is not very even by expressing that same information as 20% *unevenness* rather than 40% evenness.

There may also be some who would like a causally consistent evenness measure that is more reactive to the presence of rare types. If I attempt to derive such an evenness measure directly from the proportions, instead of following Simpson (1949) by exponentiating them first, the most obvious choice would be to scale the sum of the inverses of the proportions so that very rare types will hold extra importance for the result calculated. I think of this family as “underdog” evenness, but they are more accurately viewed as measures of the percentage of the maximum richness, which I label ^q^P_R_. They can be calculated as:

$${\;}^{q}P_{R}\equiv \left\{\begin{array}{ccc} {\left[\frac{K^{\left(q+1\right)}}{\sum_{k=1}^{K}\left(1/p_{k}^{q}\right)}\right]}^{\left(-q\right)} & , & \;q\neq 1\\ 1 & , & \;q=0\\ \frac{K}{\min(p_{k})} & , & \;q=\infty \end{array}\right.$$

This family has a number of interesting properties. First, it is highly sensitive to rare types, declining precipitously toward zero from the addition of only a few species. Second, setting the number of species K equal to 2 will make ^1^P_R_ exactly equal to ^2^D_E_, although there does not seem to be any direct correspondence between the two families for other values of K. Finally, all of the measures of the family ^q^P_R_ do not change their value under a replication transformation. As I have discussed, this replication‐invariance property is a bone of contention in the literature on evenness (Tuomisto, 2012), because it seems contrary to the intuitive behavior of evenness. While I agree with Chao and Ricotta (2019) that replication invariance is not something desirable in an evenness measure, I offer ^q^P_R_ in an attempt to propose a causally consistent, but replication‐invariant, diversity measure that is also highly responsive to rare types.

In total, then I present three families of causally consistent evenness measures that have different properties and therefore may be desirable to deploy in different settings. Table 1 summarizes these properties and indicates where each family may be of use.

**Table 1:** A brief summary of the three families of evenness measures I present

Name	Symbol	Use case
Percent evenness	^q^D_E_	A straightforward measure bounded between 0 and 1. Acceptable in most cases and interpretable as the percentage of the maximum evenness expected given the number of species present.
Evenness–unevenness index	^q^EU	Good for identifying uneven distributions in a separate category from even ones, or building face validity with nontechnical audiences.
Percent richness	^q^P_R_	Useful when you want to heavily overweight rare species in the calculation of evenness, or if you need a measure that is replication‐invariant.

## 7 ILLUSTRATING THE PERFORMANCE OF THE EVENNESS MEASURES

Figure 1 demonstrates how ^2^D_E_ and ^2^EU perform by measuring them both for example communities where K is set equal to two.

**Figure 1:** A stacked graph of proportions for eight notional communities is presented here, along with the calculated values of two evenness measures and one richness measure for *q* = 2. ^2^D_E_ is the second‐order percent evenness measure from the family ^q^D_E_. ^2^EU is the second‐order evenness–unevenness transformation. ^2^D_R_ is the second‐order Hill number, a measure focused on richness rather than evenness. The communities in this figure all have exactly two species to highlight how changes that primarily impact evenness will change the measures in question

One potential critique of ^q^D_E_ and ^q^EU might be that the absence of a species from a community is important information that we should not simply adjust away. My response to this would be to say that if a richness measure from ^q^D_R_ is going to be employed alongside of a measure from ^q^D_E_, then the information about the number of species existing in each community will still be evaluated by the study, it will just be located in the richness measure, which is the correct place for it to be reflected. I therefore report the evenness measures alongside their same order richness measure ^2^D_R_ in order to show how these two perspectives provide very different information about the diversity of each community.

If you focus on the question “roughly how many species are represented here?” ^2^D_R_ provides a good answer since it is an effective species measure. If on the other hand you focus on the question “roughly how equal in size are these species?” then it is clear that ^2^D_E_ or ^2^EU are much better choices. ^2^D_R_ may be responsive to evenness, but it does not actually communicate evenness very well, and the converse is true of ^2^D_E_.

Figure 2 reports the same three measures applied to example communities containing more than two species. This diagram highlights the way that the (*K*−1)/*K* scaling allows ^q^D_E_ to directly compare evenness across communities when the number of species changes. The large range of values of richness exhibited in these examples further shows that a single diversity measure is ill equipped to clearly communicate both richness and evenness at the same time.

**Figure 2:** A stacked graph of proportions for eight notional communities is presented here, along with calculated values of two evenness measures and one richness measure when *q* = 2. ^2^D_E_ is the second‐order percent evenness measure from the family ^q^D_E_. ^2^EU is the second‐order evenness–unevenness transformation. ^2^D_R_ is the second‐order Hill number, a measure focused on richness rather than evenness. The communities in this figure differ in the number of species present to highlight how changes that significantly alter richness will impact the three measures

Figure 3 illustrates the importance of causal consistency in the interpretation of evenness by showing ^2^D_E_ and ^2^EU alongside their causally inconsistent relative ^2^C_E_. Both ^2^D_E_ and ^2^EU respond intuitively to the test communities presented in the figure, while ^2^C_E_ is less well behaved in most cases. One particular example where the limitations of ^2^C_E_ are evident is example 3, where the community is perfectly divided between two species. Both ^2^D_E_ and ^2^EU correctly report the evenness of example 3 as 100%, but because the total number of species present between all of the example plots is nine, not two, ^2^C_E_ calculates that the evenness of example 3 is only 56%. In addition, when a single individual of a third species is added in example 4, ^2^C_E_ hardly changes, whereas ^2^D_E_ and ^2^EU are greatly reduced. This shows how the implicit assumption of all existing evenness measures, that the appropriate way to scale the evenness of a community is by expecting that community to have individuals from every species, distorts the measurement of evenness.

**Figure 3:** The stacked graph of proportions for 10 test communities is presented here, along with calculated values of three evenness measures. ^2^D_E_ is the second‐order percent evenness measure from the family ^q^D_E_. ^2^EU is the second‐order evenness–unevenness transformation. ^2^C_E_ is a causally inconsistent version of ^2^D_E_. The communities in this figure test the responses of these measures to various conceptual tests. Example 2 splits each species from example 1 in half, example 4 and 6 introduce a single individual of a rare species into the communities from example 3 and 5 respectively, example 8 reduces the dominance of the most abundant species from example 7, and example 10 reduces the number of the least abundant species from example 9

Figure 3 also confirms that the adjustments that made ^q^D_E_ causally consistent did not diminish the family's performance as an evenness measure relative to ^q^C_E_. Chao and Ricotta’s (2019) requirements that an evenness measure be continuous, invariant under changes in the ordering of proportions, Schur‐concave for cases where K is equal, and not be impacted by the units used all follow directly from the construction of ^q^D_E_ and do not need to be illustrated, but Figure 3 allows you to see examples of each of their other requirements.

Example 2 is the community that results from a replication of the species in example 1, and both ^q^D_E_ and ^q^C_E_ increase their calculation of evenness for example 2 compared with example 1. The introduction of a rare species in examples 4 and 6, compared to the perfectly even communities in examples 3 and 5, show how both ^q^D_E_ and ^q^C_E_ do not increase from the introduction of a rare species. However, these examples also show that ^q^C_E_ reduces by considerably less than ^q^D_E_, since the calculated values of ^q^C_E_ rounded to a whole number are equal in both instances. The principle of transfer is demonstrated by examples 7 and 8. Example 8 differs from example 7 in that it transfers individuals from a dominant species to a less dominant one. Both ^q^D_E_ and ^q^C_E_ follow the principle of transfer and increase in response to this change. Varying richness so much across the 10 examples also gives you a good sense of how both measures take a fixed range of values regardless of changes in richness.

## 8 CONCLUSION

There is a proliferation of competing measures of evenness, and so any new measure has a justifiably high hurdle to clear before it is accepted. I offer these three families of measures, ^q^D_E_, ^q^EU, and ^q^P_R_ in an attempt to set a new standard for measures of evenness by combining the interpretive clarity of Simpson's diversity or the Hill numbers, with the causal consistency inherent in all richness‐focused diversity measures.

The central insight that enables this innovation is a careful consideration of how the difference between the actual and potential number of species in a community impacts the evenness we should report for that community. Without adjusting for the difference between these two values, it is not possible for an evenness measure to be causally consistent, and a lack of causal consistency is neither intuitive nor desirable, especially in a controlled study.

A combination of evenness measures and richness measures is likely to be needed in order to fully appreciate the ecological impacts of diversity. ^q^D_E_ and ^q^EU both allow researchers the option to use simple, intuitive measures of evenness that are easy for their readers to understand and interpret, while remaining changeable only through changes in species abundance. Using these measures alongside a richness‐focused measure will allow diversity research to uncover more than one dimension of its many hypothesized effects.

## **CONFLICT** OF INTEREST

I declare no competing interests.

## AUTHOR CONTRIBUTION

**Kawika Pierson:** Conceptualization (lead); Methodology (lead); Visualization (lead); Writing‐original draft (lead); Writing‐review & editing (lead).

## Data Availability

This paper did not use any data. A workbook that calculates the measures reported here and generates the figures reported is available from the author.
